# Machine Learning-Based Technique for the Severity Classification of Sublingual Varices according to Traditional Chinese Medicine

**DOI:** 10.1155/2022/3545712

**Published:** 2022-11-07

**Authors:** Ping-Hsun Lu, Chih-Chi Chiang, Wei-Hsuan Yu, Min-Chien Yu, Feng-Nan Hwang

**Affiliations:** ^1^Department of Chinese Medicine, Taipei Tzu Chi Hospital, Buddhist Tzu Chi Medical Foundation, New Taipei City 23142, Taiwan; ^2^School of Post-Baccalaureate Chinese Medicine, Tzu Chi University, Hualien 97048, Taiwan; ^3^Department of Mathematics, National Central University, Jhongli District, Taoyuan City 320317, Taiwan

## Abstract

Tongue diagnosis, a noninvasive examination, is an essential step for syndrome differentiation and treatment in traditional Chinese medicine (TCM). Sublingual vein (SV) is examined to determine the presence of blood stasis and blood stasis syndrome. Many studies have shown that the degree of SV stasis positively correlates with disease severity. However, the diagnoses of SV examination are often subjective because they are influenced by factors such as physicians' experience and color perception, resulting in different interpretations. Therefore, objective and scientific diagnostic approaches are required to determine the severity of sublingual varices. This study aims at developing a computer-assisted system based on machine learning (ML) techniques for diagnosing the severity of sublingual varicose veins. We conducted a comparative study of the performance of several supervised ML models, including the support vendor machine, K-neighbor, decision tree, linear regression, and Ridge classifier and their variants. The main task was to differentiate sublingual varices into mild and severe by using images of patients' SVs. To improve diagnostic accuracy and to accelerate the training process, we proposed using two model reduction techniques, namely, the principal component analysis in conjunction with the slice inverse regression and the convolution neural network (CNN), to extract valuable features during the preprocessing of data. Our results showed that these two extraction methods can reduce the training time for the ML methods, and the Ridge-CNN method can achieve an accuracy rate as high as 87.5%, which is similar to that of experienced TCM physicians. This computer-aided tool can be used for reference clinical diagnosis. Furthermore, it can be employed by junior physicians to learn and to use in clinical settings.

## 1. Introduction

The human tongue is an essential organ of the body and can provide much information on human health status [1, 2]. Tongue diagnosis is a simple and noninvasive technique for the syndrome differentiation and treatment in traditional Chinese medicine (TCM) [3–7]. Sublingual varices are a symbol of TCM judgments of blood stasis. Furthermore, blood stasis severity can indicate disease severity related to blood stasis syndrome [8]. Sublingual varices, directly connected to internal organs through blood vessels [9], refer to the dilated veins distributed under the lateral edge of the tongue. The clinical manifestation of sublingual varices is the dilation of the small veins under the tongue. Their pathogenesis may be related to connective tissue loss or vein wall weakening with aging [10]. When healthy persons are in a sitting position, their sublingual veins (SVs) are not noticeable, and bluish-purple bands are faintly visible. However, when the central venous pressure exceeds 20 cm H_2_O, the SVs dilate and become prominent [11].

The causes of sublingual varices are not fully understood, but they may be related to age, smoking, cardiovascular disease (CVD), hypertension, and hepatocellular carcinoma (HCC) [9, 12, 13]. Zhao et al. [14] found that sublingual varices severity can be regarded as an independent risk factor for HCC, and they confirmed that the combination of alpha fetoprotein, Golgi protein 73 levels, and sublingual vein grading can accurately diagnose HCC, unlike a single parameter or a combination of two parameters. In addition, many studies have revealed that the stasis degree of the SV is closely related to disease severity. The length, width, and type of the sublingual vein patients with HCC can be used to predict changes in the inner diameter of the portal vein and hepatic artery [12]. Wang et al. [15] compared SVs of 112 patients with CVD and those of 88 healthy people without CVD as a control group. They found that the abnormal changes of sublingual vein of patients with CVD were significantly more than those in the control group, and the degree of sublingual varices is directly proportional to CVD severity. Brachial-ankle pulse wave velocity (ba-PWV) is an observation index of aortic stiffness, and it is one of the gold standards for arterial stiffness measurement [16]. When ba − PWV ≥ 1600 cm/sec, CVD is likely. In a cross-sectional study, Hsu et al. [17] demonstrated that the average ba-PWV of patients with type 2 diabetes is >1700 cm/sec, and that a higher ba-PWV corresponds to more sublingual varices severity. Sublingual varices may be related to the arterial stiffness of patients with type 2 diabetes mellitus [18]. Therefore, sublingual varices imply pathological changes in the organs, and early identification of sublingual varices severity is beneficial for early prevention and treatment. However, the inspection of sublingual collaterals is subjective. Different observers may assess the same photograph of sublingual collaterals differently [19]; hence, objective and scientific diagnostic methods are urgently required to determine sublingual varices severity.

Artificial intelligence (AI) technology can assist doctors in performing accurate diagnoses and medical image analysis to determine disease severity and reducing their workload. For example, the application of AI in liver imaging can assist in the detection and evaluation of focal liver lesions and predict the treatment response [20]. Furthermore, AI can be used to diagnose breast cancer, and it can surpass human experts in breast cancer prediction by reducing false negatives and false positives [21]. However, the method for the determination of the sublingual varices severity has not been effectively developed; most existing research works have focused on tongue surface-related topics [22–26]. This study aims at developing a computer-assisted system based on machine learning (ML) techniques to diagnose the severity of sublingual varicose veins. ML is one branch of AI techniques used for classification and prediction. The SV automatic classification system can achieve objective and quantitative data. It is hoped that this system, which uses the noninvasive SV examination approach to predict disease severity, will aid in the diagnosis and classification of diseases.

Tu et al. [27] successfully used the principal component analysis (PCA) with the sliced inverse regression (SIR) for pain prediction from electroencephalographic signals. They showed that their method is superior to the traditional dimension reduction methods, including PCA and the partial least-squares method. Furthermore, Tang et al. [25] employed the multiple-instance transfer learning-based, a popular convolution neural network (CNN) model (ResNet) for feature extraction in conjunction with a support vector machine (SVM) method for tongue coating classification. Motivated by the works of Tang et al. and Tu et al., we propose to use two model-reduction methods, PCA along with SIR and CNN to extract some valuable features from the original tongue image in conjunction with ML methods.

## 2. Materials

### 2.1. Study Population

In ML, ensuring the quality of data is crucial. Clearly labeled data can help obtain good diagnosis results in subsequent ML. The sublingual collateral images of blood stasis syndrome in this study were obtained from the Department of Traditional Chinese Medicine in Taipei Tzu Chi Hospital, from April 1, 2017 to March 31, 2022. The selection criteria were patients aged 20-80 years who received a diagnosis of the blood stasis syndrome based on the TCM technique. Patients with stroke, myocardial infarction, cancer, the Sjogren disease, chronic hepatitis, and liver cirrhosis were included, whereas those with unstable vital signs, unclear consciousness leading to an inability to communicate or severe depression or schizophrenia, or those who were pregnant or breastfeeding were excluded. The data collection and processing procedure for this study were approved by the Institutional Review Board (IRB) of the Taipei Tzu Chi Hospital (IRB number: 06-X11-029). Patient consent was obtained, and the study was conducted in compliance with the IRB regulations. The numbers of different types of diseases were as follows, 41 people with cancer, 45 people with the Sjogren disease, 3 people with systemic lupus erythematosus, 3 people with rheumatoid arthritis, 2 people with psoriatic arthritis, 1 person with hepatitis, 4 people with myocardial infarction, and 1 person with obstructive sleep apnea.

### 2.2. Image Acquisition

For obtaining photographs, the patients were asked to remain seated and roll their tongues up as much as possible for 30 seconds to expose the SV. The photographs were taken using the digital camera of a mobile phone with a forced flash. All photos were stored as 24-bit red, green, and blue (RGB) color images. Image preprocessing consisted of four steps, namely, region of interest (ROI) location, standardization, normalization, and reshaping, which convert the image to readable data for the ML methods (Figure 1). The use of the ROI as input data can increase the classification accuracy of the algorithms. A TCM physician identified the ROI and removed all irrelevant portions, such as tooth decay, dentures, or beards, from the original images. After the images were cropped, the region of each patient's tongue was placed in the middle to emphasize the SV. Because the resolution of the original photos is different, we standardize each image to a resolution of 128 × 128. We compared the ML results obtained by the images with different resolutions, ranging from 64 × 64 to 256 × 256. A preliminary study indicated a negligible difference between them, which implies that the resolution of a photo taken by a general mobile phone camera is sufficient. Finally, all imaging data sets were normalized by using the min-max scaling method to fit the range of their values between 0 and 1 to ensure the computational efficiency of the model.

The observation indices of SVs were formulated with reference to the experience of TCM physicians. Sublingual varices were classified into four levels. V1 indicates faintly visible SVs (vague type) or normal SVs; V2 indicates obvious SVs (obvious type); V3 indicates the visible branching SVs (branching type); and V4 is severely deformed vein structure, which can be seen as a bulging or bead like in series (Figure 2).

Three experienced TCM physicians in Taipei Tzu Chi Hospital independently scored the original data by examining the SV images, where V1 was scored as 1, V2 as 2, and so forth. The subjective judgment standards of each physician may be inconsistent. If the grading results determined by the physicians varied greatly, the unclear and incredible data labels would affect the accuracy rate of a ML technique.

To verify interrater reliability between the physicians, we calculated Cohen's kappa and Fleiss' kappa coefficients [28]. Cohen's kappa coefficient is used for accessing the reliability of agreement between two graders, and its range is between -1 and 1. A kappa value greater than 0.8 indicates that the agreement is almost perfect. A kappa value between 0.6 and 0.8 means substantial agreement, but a kappa value is less than 0.6 which indicates that the scoring criteria for each grader may need to be discussed again. On the other hand, Fleiss' kappa is the consistency judgment index for assessing the reliability of agreement between more than two graders, with a concept similar to that of Cohen's kappa. The closer the value to 1, the higher the consistency. Cohen's kappa values between two of the three physicians were 0.845, 0.930, and 0.879, respectively, and the Fleiss' kappa value of three physicians was 0.885. Hence, the scoring results provided by these three physicians were reliable.

For simplicity, we considered the binary classification problem, that is, the patients' sublingual varices are categorized as “mild” and “severe.” The labels (ground truths) of data used for numerical experiments were “mild”, if the average score provided by the three TCM practitioners was ≤2; it was “severe” if the average score was >2. In total, 50 images were labeled as severe and 50 as mild. The numbers of images labeled severe and mild are 50 for each case. Among the 100 patients enrolled, 87 were females, and 13 were males.

## 3. Methods

### 3.1. Available ML Techniques in Scikit-Learn

Depending on whether the ground-truth data are available as labels for training, ML methods can be classified into three categories: supervised learning, unsupervised learning, and reinforced learning. In this study, we mainly considered supervised learning techniques. In supervised learning, the data are labeled, and the machine is trained under the known ground truth. For the application of the ML technique, we divided the data set into two parts, training and testing. Training data were used to determine the method's parameters, and testing data were used to evaluate the method's efficacy. In this study, we investigated the performance of four commonly used supervised ML techniques, namely, SVM, linear regression model, decision tree, and K-nearest neighbor (KNN) and their variants, which are all available in scikit-learn, a python-based open-source package for ML [29]. In the following sections, we highlight the concepts of these methods and refer readers to references [30, 31] for details.

#### 3.1.1. Linear Regression Models

Linear regression is one of the most popular predictive methods and can also be used as a classifier. Let *y* = [*y*_1_, *y*_2_, ⋯,*y*_*m*_]^*T*^ be a label vector whose component value is either 1 or -1 for the binary classification. Here, *m* is the total number of elements in the data set. In addition, let *X* be the feature matrix, where its column vector *X*_*i*_ is the feature vectors corresponding to the *i*-th data set, given by *X*_*i*_ = [*x*_1_^(*i*)^, *x*_2_^(*i*)^, ⋯, *x*_*n*_^(*i*)^], where 1 ≤ *i* ≤ *m* and *n* is the number of features. By introducing the associate weighting vector denoted by *w* = [*w*_0_, *w*_1_, ⋯,*w*_*n*_]^*T*^, we define the prediction vector as $\hat{y}\left(w,X\right)=Xw$. The linear regression attempts to find the best weight vector such that the distance between the prediction and label vectors is minimized in the least-squares sense, i.e., find *w* such as $\min_{w}{\left\|y-\overset{\wedge }{y}\left(w,X\right)\right\|}^{2}$. In addition to linear regression, which only works for simple problems, many extended models have been developed. For example, the ridge regression adds the *α*‖*w*‖^2^ term, which can avoid a weight from having too much influence when it is too large.

#### 3.1.2. Support Vector Machines

The basic idea of SVM is try to find two parallel hyperplanes in the high-dimensional training space with a large margin as possible to separate the data points (pixels of images) into two groups based on given labels. If the data set cannot be easily classified in the original dimension, we project it to a high-dimensional space. Then, a hyperplane *w*^*T*^*x* + *b* = 0 that can separate two subsets is found. The points that determine the hyperplane are called support vectors. The distance between them and the hyperplane are the margins. SVM solves $\underset{w}{\min}1/2w^{T}w+C\varepsilon$, where *C* is a penalty coefficient to control the size of *ε*. The kernel function in SVM controls the parameters of the projection method. Common kernel functions include linear, polynomial, radical basis, and sigmoid functions. Each kernel function corresponds to a different projection method.

#### 3.1.3. Decision Trees

The training process of the decision tree technique is like building a tree diagram from top to bottom, which is composed of the root, internal, and leaf nodes. Except for the leaf nodes, all nodes representing a feature include two child nodes classified into two subgroups based on some criteria. When the feature is highly correlated with the label, it becomes a beneficial message. The main drawback of decision trees is their inaccuracy, although they are easy to implement and use. A random forest method was proposed to improve the performance of classical decision tree methods, which includes their advantages. A random forest comprises many decision trees. Although the computational cost of the random forest is high, the advantage is that it can find the best split feature and threshold value from a random subset of all features. It uses a random selection process to resolve the overfitting problem of decision trees and reduces errors through different combinations.

#### 3.1.4. Nearest Neighboring Methods

The KNN method is one of the most well-known methods in the category of lazy learning methods. In contrast to eager learning methods, such as SVMs or linear regression methods, the lazy learning method does not have any involved parameters to compute during the training step, and it only involves setting up for the classification model. For example, K-nearest neighboring data points associated with each point in the feature space are needed. During the testing phase, for this particular point, the classification of new testing data sets is decided by K-labeled nearest neighboring points, with a majority vote. The value of *K* is set to 5, and the Euclidean norm is used to measure the distance of two data points in our experiments.

### 3.2. ML Methods in Conjunction with Feature Extraction Techniques

Figure 3 presents a graphic illustration of the two proposed feature extraction processes in conjunction with ML methods, called ML-PCA + SIR and ML-CNN. In addition, the one using the original pixels of images as features is labeled as ML-original. ML stands for an ML method, for example, SVM or Ridge classifier. Feature extraction can be regarded as a process for noise removal from images. The main functions of feature extraction are to save training time and to improve the performance of ML methods.

The PCA proposed by Karl Pearson in 1901 is an unsupervised linear dimensionality reduction method and a feature extraction technique widely used in ML and statistics. Through orthogonal transformation, dependent data sets are reformulated as independent ones, and these retained data points are referred to as principal components. The basic idea of the PCA is to determine a proper lower-dimensional hyperplane such that the maximum variance is preserved. The eigenvectors (principal components) and their eigenvalues can be obtained through eigendecomposition of the covariance data matrix. The number of principal components that should be kept can be determined by computing the explained variance ratio of the data matrix. As an illustration, Figure 4 shows a comparison of the original tongue images and the recovered compressed images with different proportions of dimensions kept. For severe cases, some essential characteristics, such as visible branching veins or severely deformed vein structure, are lost if all details are not included, for example, *n* = 10 or *n* = 20 in the compressed images.

Unlike the PCA, SIR proposed by Li [32] is a nonlinear dimension reduction method of supervised learning, which requires the label *y* as an input. The critical step of SIR is to find the so-called effective dimension reduction direction initially and then project all the data into a new space, which is divided into *n* slices, where *n* corresponds to the number of categories; for example, for our target application, *n* = 2 and is based on the eigenvectors of a covariance matrix for the data where each slice is located. It is different from the PCA in that all the data are generated together to perform the dimension reduction action. The projection direction is determined using PCA. One constraint of SIR is that this technique requires the number of samples to be greater than the number of features. Therefore, as suggested by [27], we apply PCA first to meet the requirement of SIR before SIR employed.

In addition, the CNN in deep learning, which is a powerful technique for image classification, can be used for feature extraction in conjunction with ML methods. CNN mainly consists of a convolution layer, pooling layer, flattening process, and fully connected layer (bottom of Figure 3). First, the primary role of the convolution layer is to extract features. A kernel convolutes with the image matrix to generate a corresponding feature map. Different kernels produce different feature maps. The automatic extraction of diversified features by using different kernels is an advantage of deep learning over ML. Second, the max-pooling method is applied in the pooling layer if the largest value in the matrix is extracted. The other alternative options are the average pooling and minpooling methods. We generate many feature maps after passing through the convolution and pooling layers. Third, the flattening process transforms our feature maps into a one-dimensional vector to form a neural network architecture. Lastly, the fully connected layer is similar to a neural network. The nodes of each layer are connected to all nodes of the next layer. A weight associated with two nodes reflects the importance of the message represented by the previous node to the next node. Instead of the predicted result, the nodes in the fully connected layer are output as features.

### 3.3. Experimental Design

The number of data sets for the current study is somewhat limited; hence, the results obtained by one particular training and testing set may not necessarily represent the learning results. Therefore, we used cross-validation to enhance the credibility of our diagnostic system; the cross-validation method can evaluate the quality of the model and its generalization ability accurately and avoid model overfitting. In particular, we used k-fold cross-validation, where the original data are divided into *k* subgroups to ensure that the number in each one is roughly the same to avoid the problem of ML tendencies caused by unbalanced data. The original data set is divided into *k* subgroups randomly. Then, one subgroup at a time is taken for testing, and the remaining *k* − 1 subgroups are used to train the model. We repeat the same procedure *k* times until each subgroup is tested. In the numerical experiment, the number of folds, *k*, is chosen to be 5. For the CNN-based feature extraction method, we use 64 of the 80 data points as the training set and remaining data points as the validation set. Its architecture is built and implemented by Keras [33], a python-based deep learning application programming interface. In the iterative process of CNN, the weights are adjusted according to the validation set results, and 40 iterations are performed for training the CNN model. Trained 1000 nodes in the middle of the fully connected layer are used as features for ML methods. A python package, namely, “sliced” [34] for SIR along with the PCA routine in scikit-learn, is used as the feature extraction tool in our study. All numerical results reported in the next section are obtained by performing a 5-fold validation four times.

## 4. Results

### 4.1. Learning Model Selection

Table 1 summarizes the mean accuracy with 95% confidence intervals (CI) and training time for the selected supervised classifiers available in scikit-learn, which are used for numerical experiments in this study. No parameter tuning is performed, and the default values for each scikit-learn classifier can be found on the website of scikit-learn [29]. The accuracy for binary classification problems [31, 35] is defined as Accuracy = (TP + TN)/(TP + TN + FN + FP), where true-positive (TP) means the presence of a disease correctly predicted; true-negative (TN) means the absence of a disease correctly predicted; false-positive (FP) means that a disease is predicted, but it is absent, and false-negative (FN) means a disease is predicted to be absent but is present. For each ML method, we included the results obtained using the original pixels and the features extracted using PCA with SIR and CNN techniques, respectively. For SVM, we included two types of kernel functions, linear and radial basis functions (RBFs). Two linear regression type classifiers with or without penalty parameters added were considered, corresponding to the ridge and linear regression, respectively. In addition, three methods, namely, decision tree, random forest, and KNN methods were included.

When the original image was used, the performance of SVM and linear regression type classifiers was comparable (84.7% vs. 84.8%), and both classes of methods outperformed the KNN (76.2%) and decision tree methods (67.7% and 75.5% for random forest). The classification problem is linearly separable. As a result, the SVM with the linear kernel is sufficient; no apparent advantages of using nonlinear kernel functions were observed, such as radial basis and polynomial functions. Similarly, the accuracy values of the linear regression and Ridge classifiers were similar (84.8% and 84.7%, respectively). On the other hand, the random forest (75.5%) outperformed the decision tree (67.7%).

For PCA dimension reduction, we tested the ML methods with different dimensions of the features kept based on the explained variance ratio, ranging from 77% to 99%, which corresponds to the reduced dimension from *n* = 10 to *n* = 87. The accuracy of ML increased by at least 10% as the explained variance ratio increased by up to 90%; then, it became insensitive in the range of 90% to 99%. The second column of Table 1 shows 95% CI values. We found that the mean accuracy of almost ML-PCA approaches was close to that of ML-original, except for the one with decision tree. With SIR in conjunction with PCA, all ML methods achieved almost the same level of mean accuracy, that is, approximately 83.5%-84.5%. The last column of Table 1 presents the result obtained using CNN for feature extraction with ML methods against the results obtained using the ML-original method. CNN could improve the diagnostic ability of most ML models, particularly for decision tree (by approximately 10%) and random forest (by approximately 8%).

### 4.2. Diagnostic Performance Comparison of ML Methods with the Results of TCM Doctors

Table 2 provides the diagnostic performance of two ML techniques in conjunction with three feature extractions, compared with the results determined by two TCM doctors, who were different from three TCM doctors in charge of determining the ground truths for experiments. Furthermore, the training times for each case are also included in the table. In the binary classification problem, in addition to accuracy, the commonly used metrics for performance evaluation are the sensitivity, specificity, positive predictive value (PPV), and negative predictive value (NPV) [31, 35], where these metrics are defined as follows. Sensitivity = TP/(TP + FN), Specificity = TN/(FP + TN), *P*PV = TP/(TP + FP), and NPV = TN/(TN + FN). Furthermore, the receiver operating characteristics (ROC) curve and the corresponding area under the curve (AUC) are valuable tools for assessing the performance of the proposed methods [29, 31, 35]. The significant difference for classification between the ML methods and TCM doctors was tested by a two-sample *t*-test. The result was considered statistically significant if the *p* value < 0.05.

The accuracy of these six methods ranged from 84.5% to 87.5% with no noticeable difference. The highest accuracy was achieved by Ridge-CNN (87.5%), which was not a statistically significant difference from that of the TCM doctors (90.0% and *p* = 0.26110). For sensitivity, SVM-CNN and Ridge-CNN were comparable (91.0% and 90.5%), and their corresponding *p* values versus the TCM doctors were *p* = 0.29190 and *p* = 0.25696, respectively. In addition, the CNN-type feature extraction for SVM or the Ridge methods exhibited sensitivity increased by approximately 10% compared with the other alternatives, including SVM-original, Ridge-original, SVM-PCA + SIR, and Ridge-PCA + SIR. The sensitivity of these four methods was lower than that of the TCM doctors, whose *p* values all are ≤0.05. Similarly, for NPV, SVM-CNN and Ridge-CNN (91.2% and 91.3%) were better than the other four methods with their values ranging from 82.1% to 83.3%, and there are no statistically significant differences versus those of the TCM doctors (*p* = 0.20108 and *p* = 0.23397). In addition, the specificity and PPV of Ridge-original were the highest among all ML methods, although the *p* values of these six methods against the TCM doctors were all ≥0.05.

For timing results, PCA + SIR feature extraction techniques can save a tremendous amount of training time for SVM or Ridge classifiers, with the speedup in a magnitude of approximately two or three orders. By contrast, because the dimension of features extracted from CNN is larger than the one obtained from PCA + SIR and the computational cost for building the CNN model is more than that for PCA + SIR, the speedup for SVM or the Ridge classifiers is less significant, 378.0 and 41.0, respectively.

Figure 5 shows the ROC analysis and corresponding AUC for four selected ML methods, including SVM (linear), Ridge classifier, KNN, and Random forest with different features. The original image and features extracted by PCA + SIR and CNN were used for ML. The corresponding AUC for each case is also presented in the figures. When the original image is used, the values of AUC for SVM and Ridge classifier are higher than KNN and Random forest (0.92 (or 0.93) versus 0.83 (or 0.82)). On the other hand, when PCA + SIR or CNN extracted the features, we can see no significant difference in AUC for the four methods, ranging from 0.88 to 0.95, which indicates that both methods effectively extracted features or removed noises from the original images.

## 5. Discussions and Conclusions

The purpose of this study was to develop an AI technique-based application for classifying the severity of sublingual varices. SV examination is a simple and noninvasive technique unique to TCM. Many studies have shown that the severity of SV stasis positively correlates with disease severity. One of the essential features of our proposed tool is the ability to use images of the SV obtained using an ordinary mobile phone or digital camera so that even nonprofessionals can efficiently use it for prescreening purposes to reduce TCM physicians' workload. Some similar works have been conducted with a focus on the tongue surface. For example, Hu et al. [36] photographed the tongue surface with a mobile phone and used the SVM-based lighting condition estimation method and ColorChecker for color correction. Their study revealed that the shape and fur of the tongue have a strong correlation with aspartate aminotransferase and alanine transaminase levels. Alternatively, some researchers have used hyperspectral images [37–39], for which specific devices were used. For instance, Li and Liu developed algorithms to extract critical features such as color [37] and fissure [39] from the hyperspectral images of the tongue surface.

In this study, we focused on evaluating the performance of the ML method, which will serve as the kernel of a diagnosis application tool. Some images include tooth decay, dentures, beards, or other irrelevant parts, which lead to ML classification errors. Therefore, ROI positioning is crucial in the preprocessing phase compared with standardization and normalization. No sophisticated automatic segmentation technique is needed to extract sublingual collaterals, such as varicose, branch, columnar, and bubbly veins [40]. Remarkably, the ROI location step can increase the accuracy of ML methods by 20%, with an improvement from approximately 60% to 80%. In addition, we recommend using RGB color images rather than the greyscale format to prevent the loss of essential information needed for the classification (65% vs. 80%).

We conducted an intensive numerical experiment to select a suitable ML model after testing all ML models available in scikit-learn and reported the comparison results of four representative classes of methods in Table 1, obtained using hypermeters with default values associated with the ML models. Selection criteria included the mean accuracy, variance, and timing for training. On the basis of results shown in Table 1, we recommend the Ridge classifier and SVM with linear kernel because of their high mean accuracy, low variance value, and less training time.

In conclusion, with the help of these two extraction methods, PCA + SIR and CNN, the training speed of the ML method can be increased by at least 40 times compared with the method that used the original image as training features, and the accuracy rate for Ridge-CNN is as high as 87.5%, which is close to that of experienced TCM doctors. This computer-aided tool can be used for reference clinical diagnosis and for learning and use by junior physicians.

## Figures and Tables

**Figure 1:** Major steps in the data preprocessing. (a) ROI identification, (b) standardization, (c) normalization, and (d) reshaping.

**Figure 2:** the typical four-level classifications of sublingual varices. We confine our study to the binary classification problem, that is, V1 and V2 were classified as “mild”; whereas, V3 and V4 were classified as “severe.”

**Figure 3:** In addition to the original standard ML, a graphic illustration for two proposed feature extraction process in conjunction with ML methods.

**Figure 4:** Comparison of the original tongue images (left column) and the one recovered from the compressed data with different proportions of dimensions retained (right column) for mild and severe cases.

**Figure 5:** The ROC analysis and corresponding AUC for selected MLs with different features. Left: original images; middle: the feature extracted by PCA + SIR; right: the one extracted by CNN. Four ML methods are considered: SVM (Linear), Ridge classifier, KNN, and Random forest.

**Table 1:** A comparison of different ML methods by using features extracted with PCA + SIR or CNN methods as well as the original images. The numbers in the table are the mean accuracies in %, and The number in square brackets is the 95% CI. Training time measured in seconds.

MLs	ML-original (%)	ML-PCA (%)	ML-PCA + SIR (%)	ML-CNN (%)	Time (s)
SVM (RBF)	78.0 [74.7-81.3]	79.0 [76.3-81.7]	83.8 [81.0-86.5]	80.7 [77.5-84.0]	11.7
SVM (linear)	84.5 [81.6-87.4]	83.3 [79.1-87.4]	83.5 [79.8-87.2]	86.2 [82.8-89.7]	40.2
Linear model	84.8 [82.0-87.5]	84.5 [81.5-87.5]	84.5 [81.5-87.5]	83.5 [79.5-87.5]	2.2
Ridge classifier	84.7 [82.3-87.2]	85.0 [81.9-88.1]	84.5 [81.5-87.5]	87.5 [83.8-91.2]	1.6
KNN	76.2 [72.5-80.0]	76.8 [73.2-80.3]	84.0 [80.9-87.1]	82.0 [79.0-85.0]	8.9
Decision tree	67.7 [61.6-73.9]	60.5 [55.8-65.2)	83.8 [80.3-87.2)	77.8 [74.7-80.8]	14.4
Random forest	75.5 [71.3-79.7]	73.2 [69.3-77.2]	83.8 [80.3-87.2]	83.8 [81.1-86.4]	21.4

**Table 2:** Diagnostic performance summary of two ML techniques in conjunction with two feature extraction techniques by using original images as features, compared with the diagnoses by two TCM doctors. The number in square brackets is the 95% CI. For each case, training time is in seconds including the time spent by a feature extraction technique when applied. The numbers in parentheses are speedup for the counterpart method against the one trained with original features.

	Sensitivity (%)	Specificity (%)	Accuracy (%)	PPV (%)	NPV (%)	Time (s)
TCM doctors	94.5 [90.3, 98.7]	85.5 [80.6, 90.4]	90.0 [87.3, 92.7]	87.6 [83.7, 91.5]	94.9 [91.2, 98.5]	N/A
SVM-original	80.5 [74.5, 86.5]	88.5 [84.4, 92.6]	84.5 [81.6, 87.4)	88.3 [84.7, 91.9]	83.1 [78.8, 87.5]	3.8e1 (1.0)
Ridge-original	79.5 [74.1, 84.9]	90.0 [86.6, 93.4]	84.7 [82.3, 87.2]	89.7 [86.4, 93.0]	82.3 [78.8, 85.8]	1.1e0 (1.0)
SVM-PCA + SIR	79.0 [72.1, 85.9]	88.0 [84.1, 91.9]	83.5 [79.8, 87.2]	87.2 [83.5, 90.9]	82.1 [77.2, 87.0]	1.8*e* − 2 (2100.0)
Ridge-PCA + SIR	81.0 [75.1, 86.9]	88.0 [84.7, 91.3]	84.5 [81.5, 87.5]	87.5 [84.4, 90.6]	83.3 [79.0, 87.7]	4.0*e* − 3 (275.0)
SVM-CNN	91.0 [85.5, 96.5]	81.5 [76.4, 86.6]	86.2 [82.8, 89.7]	83.8 [80.0, 87.6]	91.2 [86.5, 95.8]	1.0*e* − 1 (378.0)
Ridge-CNN	90.5 [84.5, 96.5]	84.5 [78.7, 90.3]	87.5 [83.8, 91.2]	86.5 [82.1, 90.9]	91.3 [86.4, 96.2]	2.7*e* − 02 (41.0)

## Data Availability

The data utilized to support the findings of this study are included in the article.
